# Real-Time Control of Intelligent Prosthetic Hand Based on the Improved TCN

**DOI:** 10.1155/2022/6488599

**Published:** 2022-05-14

**Authors:** Xiaoguang Liu, Jiawei Wang, Tingwen Han, Cunguang Lou, Tie Liang, Hongrui Wang, Xiuling Liu

**Affiliations:** ^1^College of Electronic and Information Engineering, Hebei University, Baoding, Hebei, China; ^2^Key Laboratory of Digital Medical Engineering of Hebei Province, Hebei University, Baoding Hebei, China

## Abstract

Intelligent prosthetic hand is an important branch of intelligent robotics. It can remotely replace humans to complete various complex tasks and also help humans to complete rehabilitation training. In human-computer interaction technology, the prosthetic hand can be accurately controlled by surface electromyography (sEMG). This paper proposes a new multichannel fusion scheme (MSFS) to extend the virtual channels of sEMG and improve the accuracy of gesture recognition. In addition, the Temporal Convolutional Network (TCN) in deep learning has been improved to enhance the performance of the network. Finally, the sEMG is collected by the Myo armband and the prosthetic hand is controlled in real time to validate the new method. The experimental results show that the method proposed in this paper can improve the accuracy of the control intelligent prosthetic hand, and the accuracy rate is 93.69%.

## 1. Introduction

In many areas, intelligent prosthetic hands can replace humans to complete the work, such as intelligent prosthetic hands instead of human remote completion of dangerous tasks and intelligent prosthetic hands to assist human rehabilitation training. But in the complex and changing environment, the traditional control of intelligent prosthetic hand method gradually cannot adapt to the requirements. In order to control the intelligent prosthetic hand efficiently and accurately, this paper adopts a human-computer interaction control method based on sEMG. This method can directly react to the human movement intention and control the intelligent prosthetic hand more accurately.

The sEMG is a bioelectrical signal generated by the contraction of muscles on the surface of the body. It is a nonstationary electrical signal with a weak amplitude of 0-1.5 mV [1]. However, sEMG contains rich information relevant to movement [1, 2]. With the in-depth study and the rapid development of bioelectrical signal detection technology, sEMG signals have become widely used, such as for the myoelectric controlled prosthesis wheelchair [3] and assistive robots [4]. Meanwhile, gesture recognition is used in remote rescue [5] and factory robots [6]. Using sEMG to control exoskeleton robots and intelligent prosthetic hands can help people accomplish dangerous tasks remotely and also assist people in rehabilitation training. Therefore, sEMG-based human-robot interaction has become a hot research topic.

For traditional machine learning methods, the accuracy of gesture recognition is low when the raw sEMG signals are used as input data [7]. Therefore, researchers considered the use of data processing and analysis. Hudgins et al. designed a feature set, containing zero crossings (ZC), slope sign changes (SSC), mean absolute values (MAV), and waveform lengths (WL) [8]. Khushaba et al. introduced a novel feature set containing seven time-domain descriptors for the extraction of spatiotemporal information [9]. Also, Tang et al. combined image entropy and density clustering to exploit the keyframes from hand gesture video for further feature extraction [10]. Image processing methods are discussed in [11] which contribute to better feature extraction.

In this domain, classification methods can be divided into machine learning and deep learning approaches [12]. Researchers have tried a variety of approaches to attain a high classification accuracy (CA). Now, conventional machine learning classifiers include Support Vector Machines (SVMs), Linear Discriminant Analysis (LDA), and *k*-Nearest Neighbors (KNN) [13–16]. Convolutional Neural Network (CNN) and Recurrent Neural Network (RNN) are the most popular deep learning algorithms for image processing [17–21]. Panagiotis et al. [22] applied TCN to gesture recognition based on sEMG, in which the output layer of TCN was further processed through average over time (Aot) or an attention (Att) mechanisms so that the complete sequence could be described by the use of tag like.

The main contribution of our work is proposed a new multichannel fusion scheme and the improved TCN structure. The MSFS method improves the accuracy of gesture recognition without increasing the number of electrodes, and this method can improve the portability of signal acquisition equipment. The core idea of this method is to increase the number of channels of the sEMG signal virtually with a limited number of sEMG electrodes. Finally, this paper constructed an online control system for intelligent prosthetic hand. The scheme of this paper is shown in Figure 1. In Figure 1, Myo_data is collected data using Myo armband; ML is machine learning; TCNS and TCND are the improved TCN structure.

## 2. Materials and Methods

### 2.1. Experimental Setup and Protocol

The data recorded in the Myo dataset came from 10 healthy volunteers, and these data were collected by the Myo armband (referred to as the Myo_data in this paper). The details of the volunteer information are shown in Table 1.

The subjects are asked to not exercise vigorously before the experiment to avoid the effects of muscle fatigue [23]. Before wearing the Myo armband, body hair is removed from the measuring area, and the skin was wiped with 75% alcohol. During the entire process of sEMG acquisition, every volunteer must wear the Myo armband in the same position. The logo LED of the Myo armband and the middle finger of the subjects are aligned.

During the data collection process, each volunteer was asked to imitate 10 gestures with the right hand, and each gesture was repeated 6 times.  Figure 2 graphically shows each gesture, with the names of the ten different gestures in the figure: (a) no. 1, (b) no. 2, (c) no. 3, (d) no. 4, (e) no. 5, (f) no. 6, (g) first, (h) good, (i) correct, and (j) okay. Each repetition lasts for 3 (or 6) seconds, and the rest for 5 seconds after the action. The Myo armband has eight sEMG differential electrodes and a 9-axis inertial measurement unit (IMU). It provides a sampling frequency of 200 Hz [22]. Before the experiments, participants were informed and filled out a written informed consent form. The study was conducted in accordance with the Declaration of Helsinki, and the protocol was approved by the Ethics Committee with reference (HDFY-LL-2020-091).

Four of these ten subjects were selected for testing in the experiment of real-time gesture recognition. The preparation process and gestures before data acquisition were as described above. Four subjects were able-bodied and free of any muscular disorders, and the specific information of the subjects is shown in Table 2.

### 2.2. Multichannel Fusion Method

The more data acquisition channels, the richer the action information it contains. At the same time, as the number of data channels increases within a certain range, the accuracy of gesture recognition will increase [24]. Therefore, this paper proposes a new channel fusion algorithm that can virtually increase the number of channels and improve the gesture recognition accuracy.

In this work, we use a two-dimensional array (*s* ∈ array(*m* × *N*)*S* ∈ array(*m* × *N*)) to represent the sEMG signals, as the input data of MSFS, where *s* represents the data of a hand movement in a single experiment, *m* (an even number) is the number of samples for each channel, and *N* is the number of channels in the array.

The operation of MSFS consists of three stages, including sample decomposition, sample reorganization, and data fusion. The details are shown in Figure 3.

In the sample decomposition process, by splitting the sEMG data by rows, we can get *m* sEMG samples of size (1 × *N*), as

(1) $$\begin{array}{c} s_{i}=\left\{s_{1},s_{2},\cdots ,s_{m-1},s_{m}\right\}, \end{array}$$

where *s*_*i*_ represents the decomposed samples and *i* is the label of the samples. In the sample reorganization stage, we recombine *s*_1_, *s*_3_, *s*_5_, ⋯, *s*_*m*−1_ into data block *A* and recombine *s*_2_, s_4_, s_6_, ⋯, s_*m*_ into data block *B*. The size of data block *A* and *B* is ((*m*/2) × *N*); Equations (2) and (3) show the structure of the data.

(2) $$\begin{array}{c} A=\left\{s_{1},s_{3},s_{5},\cdots ,s_{m-1}\right\}, \end{array}$$

(3) $$\begin{array}{c} B=\left\{s_{2},s_{4},s_{6},\cdots ,s_{m}\right\}. \end{array}$$

In the data fusion stage, we spliced the two data blocks (*A*, *B*) into data block *C*. The size of data block *C* is ((*m*/2) × 2*N*); its structure refers to (4). The specific operation of MSFS is shown in Figure 3. In Figure 3, *s*_*i*_ represents the samples of the original sEMG signals; *m* represents the number of samples; *N* represents the number of channels, and 2*N* represents the number of virtual channels.

(4) $$\begin{array}{c} C=\left\{s_{1},s_{3},\cdots ,s_{m-1},s_{2},s_{4},\cdots ,s_{m}\right\}. \end{array}$$

Adjacent samples of *s*_*i*_ possess similarity (like *s*_1_ and *s*_2_ and *s*_2_ and *s*_3_). After MSFS, the nonadjacent samples have the chance to get closer (like *s*_1_ and *s*_3_ and *s*_2_ and *s*_4_), which could reveal hidden correlations between nonadjacent samples. On the other hand, *s*_1_ and *s*_2_ are fused into a new sample, which is equivalent to the fusion of two samples with high similarity for parallel processing. In this operation, raw sEMG signals are stacked row by row into a data block (Figure 3 (block A and block B)) based on algorithm MSFS. Then, the two data blocks (data block *A* and *B*) are concatenated into data block *C*(Figure 3 (block C)). Finally, the input data (*m* × *N*) become data block *C*((*m*/2) × 2*N*), and the number of channels is increased from *N* to 2*N*.

In order to study the performance of the reorganization fusion structure, this paper records the absolute value of the average Pearson correlation coefficient |*r*| between adjacent rows (adjacent columns) data before and after using the reorganization fusion algorithm, as shown in Table 3. The above correlation coefficient satisfies the significance condition and has statistical significance. A high correlation coefficient indicates a high degree of similarity between data and the more similar the hand movement information contained. On the contrary, the lower the value, the more diverse the information contained.

It can be seen from Table 3 that whether it is between adjacent rows or adjacent columns, the correlation of the signal before MSFS processing is greater than the signal after MSFS processing. It can be inferred from this that the MSFS algorithm can reduce the correlation between the data and make the data characterize more abundant and effective hidden hand movement information, which is beneficial to the subsequent signal analysis and feature extraction.

### 2.3. Data Preprocessing and Feature Extraction

The regular frequency of the sEMG signals generated from gesture execution ranges from 20 Hz to 500 Hz [25]. In this paper, the third-order Butterworth bandpass filter is used to retain signals with frequencies between 20 Hz and 200 Hz. The attenuation rate of the filter is 18 dB per octave. At the same time, this paper uses a notch filter to remove 50 Hz power frequency interference. In order to prove the effectiveness of the filter, Figure 4 shows the comparative spectrogram before and after sEMG filtering.

Before feature extraction, the sliding window strategy is utilized for the segmentation of the sEMG signals to ensure the continuity of features. The data is divided into windows by a sliding window strategy to determine the features. We use (5) to calculate the number of windows:

(5) $$\begin{array}{c} W=\frac{n-\text{window}\_\text{size}}{\text{sliding}\_\text{step}\_\text{size}}+1, \end{array}$$

where *W* is the number of windows and *n* is the sample-point number of the sEMG. The operation of the sliding window is shown in Figure 5.

In order to ensure that the experimental comparison is carried out fairly, sEMG inputs with the same total sample size are selected for both types of experiments, and two types of window sizes are set in this paper according to whether the MSFS algorithm is used to process the signals. The first size is for the no MSFS experiment (window size is 1000 ms, the sliding step is 100 ms, and the data is updated every 100 ms); the second is the MSFS experiment (window size is 500 ms, the sliding step is 50 ms, and the data is updated every 100 *ms*). In both methods, the total amount of data in each window and the total amount of data in the sliding step are equal. In general, delays of 300 ms or less are acceptable for real-time control, and segments that are too long could hinder real-time operation [26]. In this paper, the data is updated every 20 points that means the data segmentation is updated every 100 ms and the time delay is acceptable.

At present, the commonly used feature extraction methods in sEMG-based application systems include time-domain feature methods, frequency-domain feature methods, and time-frequency domain feature methods [27]. From the perspective of comprehensive consideration, this paper constructed a feature set to extract features of sEMG and it could obtain richer gesture characterization information. This feature set includes the above-mentioned 8 types of time domain features and 2 types of frequency domain features, including mean absolute value (MAV), root mean square (RMS), standard deviation (STD), waveform length (WL), Willison amplitude (WA), zero crossing (ZC), sign change of slope (SSC), integrated electromyogram (IEMG), mean power frequency (MPF), and median frequency (MF).

The calculation of the feature set can provide rich information for the classification of hand movements, and at the same time, it will also lead to a rapid increase in data dimensions. High-dimensional input data is prone to dimensional disasters, which invisibly increases the requirements for the memory and processing capabilities of the computing system and affects the recognition effect of the classifier's hand movements. Therefore, it is also necessary to reduce the dimensionality of the data after feature extraction, which will be discussed in Experimental Results and Discussion of this paper.

### 2.4. Gesture Recognition Proposed Method

The TCN includes convolutional layer, residual connection, and fully connected layer. Among them, the convolutional layer uses the dilated convolution operation method. The dilated convolutional layer is a unidirectional structure, and the structure flow of this layer is shown in Figure 6.

After several comparison tests, the parameter values chosen in this paper are dilated coefficient *d* = 2, convolution kernel size *k* = 3, convolution stride = 1, padding = SAME, and the receptive field of neuron is 5. The input data size of the TCNS and TCND is (21 × *n*), where *n* is the dimension of the input data and 21 is the number of samples. This paper uses single-dimensional data (21 × 1) as an example to illustrate the network architecture.

#### 2.4.1. Temporal Convolutional Network-Single (TCNS)

The network structure of TCNS is shown in Figure 7. The network includes TCNS_1 and TCNS_2 substructure blocks, residual connection, and full connection layer. Both substructure blocks include two dilated convolutional layers, and there is a batch normalized BN layer between each dilated convolutional layer and the activation layer.

The residual structure connects the initial input information of the entire network with the feature data output by the hidden layer, which can effectively alleviate the problem of network degradation. After the training is completed, the data is tiled and input into the fully connected layer, and the number of classification results output by the last fully connected layer is the same as the number of gestures to be classified. The dilated coefficient *d* in this structure increases with the deepening of the network, which can increase the receptive field of neurons and gradually obtain more global hand motion characterization information.

#### 2.4.2. Temporal Convolutional Network-Double (TCND)

The structure of TCND is shown in Figure 8. The network consists of two channels, each of which includes three dilated convolutional layers and one residual structure, and there has one BN layer between each dilated convolutional layer and the activation layer.

In this structure, the TCND_1 channel *d* = 2, the receptive field of the network neuron is small, that is, the convolution operation is performed in a small range to extract the relatively detailed action characterization information in the input data. TCND_2 channel *d* = 4, relative the receptive field of the TCND_1 channel neuron is enlarged, that is, more global information can be obtained. After the fusion of the two channels of information, the TCND network has more diversified gesture representation information, which helps to improve the classification results.

## 3. Experimental Results and Discussion

In order to verify the effectiveness of the method proposed in this paper, two cases of offline gesture recognition and real-time gesture recognition are verified. Experiment 1 and Experiment 2 are offline gesture recognition experiments, and DB5 database (DB5 is the fifth subdataset of the publicly available multimodal database, and the dataset records sEMG for 10 complete subjects) with Myo_data is selected as the experimental data. The effect of MSFS algorithm is verified by experiment 1 through experimental comparison. Experiment 2 verifies the gesture recognition accuracy of TCNS and TCND network structure. Experiment 3 is a real-time gesture recognition experiment, through which the sEMG of 10 gestures of the subject is collected in real time, and the subject's own network model is constructed and the accuracy of gesture recognition is verified.

### 3.1. PCA-Based Feature Information Optimization

The calculation of the feature set can provide rich information for the classification of hand movements, and at the same time, it will also lead to a rapid increase in data dimensions. High-dimensional input data is prone to dimensional disasters, which invisibly increases the requirements for the memory and processing capabilities of the computing system and affects the recognition effect of the classifier's hand movements.

This paper chose to use the Principal Component Analysis (PCA) to perform dimensionality reduction and feature selection on the high-dimensional data after feature extraction and select the retained feature dimensions by comparing the cumulative variance contribution rate of each input data. As shown in Figure 9, for the Myo_data database, the number of channels of the original sEMG is 8. After feature extraction, an 80-dimensional feature vector is obtained.

Shown in Figure 9(a) is the cumulative variance contribution of 10 components. The rate has reached more than 95%, so the first 10 principal components are selected as the best dimensionality reduction result.  Figure 9(b) shows that the top 20 principal components are selected as the best dimensionality reduction results using the MSFS method of Myo_data.  Figure 9(c) shows that the DB5 database selects the top 20 principal components as the best dimensionality reduction result.  Figure 9(d) shows that DB5 using MSFS method selects the first 40 principal components as the best dimensionality reduction results. The dimensionality reduction results of each database are shown in Table 4.

#### 3.1.1. Gesture Recognition Based on Machine Learning (Experiment 1)

Experiment 1 used three machine learning algorithms: KNN, LDA, and SVM to recognize gestures. This paper used the cross-validation method when calculating the indicators of gesture recognition. Specifically, the data of each gesture is divided into 10 parts, each part in turn as the test set, and the rest as the training set. The final experimental result is the average of 10 cross-validation. In this paper, accuracy, recall, and precision are used to evaluate this system, and Table 5 shows the results.

The three algorithms in this experiment are all constructed by the scikit learn library in Python 3.7, and the ratio of training set to test set is 1 : 9. In this experimental results below, Y indicates that the MSFS algorithm is used, and N indicates that the MSFS algorithm is not used.

According to the experimental results, the MSFS method based on sEMG has excellent performance for recognizing hand gestures. The effect of gesture recognition based on KNN and LDA is equivalent, and the average accuracy and other indicators have reached more than 87%. At the same time, the MSFS algorithm also played a role in this experiment.

The accuracy of the classifier is the most common evaluation criterion, which visually reflects the probability of predicting a correct gesture. In this paper, recall, precision, and *F*1 score are added as auxiliary evaluation metrics. According to the experimental results, the *F*1 score for LDA with KNN using the MSFS method is higher than the method without MSFS.

#### 3.1.2. Gesture Recognition Based on TCNS and TCND (Experiment 2)

Experiment 2 used TCNS and TCND to recognize 10 gestures. Parameters of TCNS: the size of the convolution kernel of the dilated con_1 (2, 4, and 5) is *k* = 1 × 3; stride = 1; padding = SAME; the values of the convolution layer *d* are set to 1 (2, 4, and 8). Each of the two residual block structures contains 1 convolution layer with dilated factor *d* = 1; the convolution kernel size of this layer is *k* = 1 × 1; stride = 1; padding = SAME.

Parameters of TCND: the size of the convolution kernel of the dilated con_1 (2, 4, and 5) is *k* = 1 × 3; stride = 1; padding = SAME; the TCND_1 part has two *d* = 2 dilated convolutional layers, and the TCND_2 part is the two dilated convolution layers. Then, the output fusion of the above two channels is combined by applying the dilated con_7 and dilated con_8.

Table 6 shows the average accuracy of gesture recognition based on TCNS and TCND.

This experiment uses the visualization tool TensorBoard provided by TensorFlow to optimize the network model. The training results of the TCNS and TCND network using the MSFS algorithm are shown in Figure 10.

As the number of network training steps increases, the gesture recognition accuracy of the two network structures gradually increases. Before the number of training steps reaches 10, the recognition accuracy of the two increases quickly, and then, the accuracy rate is in a steady upward trend. By observing the accuracy curves of the training set, it can be found that when the number of training steps is more than 30, and the accuracy curves of the training sets of the two networks gradually become stable. In the training process of TCNS and TCND network, the program will save the model parameters of the corresponding network and apply the training results to subsequent network test experiments.

Figure 11 shows the loss change curve of the corresponding network.

When the training steps are less than 20, the loss curves of the two network structures are in a state of rapid decline, but it can be clearly observed that the loss curve of the TCND network declines faster. In addition, the loss curves of the training set of the two networks fluctuated between 50 and 60 steps. Among them, the fluctuation amplitude of the TCNS network is larger than that of TCND. By analyzing the curve of the accuracy and loss of the above network training set, it can be found that the gesture recognition effect of the TCND network is good and relatively stable.

The comparison of Figure 12 shows that the recognition accuracy of the TCN is relatively high, and the classification effect of the TCND network is significantly higher than the other four classification algorithms. Moreover, the performance will be more superior when adapted MSFS method. Therefore, this paper used TCND network for real-time gesture recognition.

#### 3.1.3. Online Gesture Recognition and Prosthetic Hand Control (Experiment 3)

The intelligent prosthetic hand interaction system based on sEMG is composed of three parts: sEMG collection, gesture recognition, and intelligent prosthetic hand control.

The prosthetic hand used in this study is made by 3D printing technology. The 3D printing material used in the smart artificial hand is a nylon material made of polyamide resin. The structure of the prosthetic hand includes five fingers, a palm, and a base, and the components are connected by 11 SG90 servos with an angle ranging from 0 to 180 degrees. Different gestures correspond to different finger bending states, and the bending and extension of the fingers depend on the change of the rotation angle of the steering gear. The hardware structure of prosthetic hand control system is shown in Figure 13.

The implementation process of the system is shown in Figure 14.

Experiment 3 included 4 of the 10 subject groups; they are healthy and without any muscle diseases. This experiment consists of two stages. The first stage is the network model training stage. The experiment subjects need to make 10 gestures in the prescribed order (the gestures are the same as the Myo_data database). Each gesture lasts for 5 s, and there are 5-second rest time between different gestures, the above experiment procedure needs to be repeated for 20 rounds, and there is a 5-minute rest time between each round of experiments. At this stage, the sEMG data collected by each subject will be stored separately, and then, network training will be carried out separately and the subject's own network model will be constructed.

The second stage is the online test stage. In this stage, the above-mentioned subjects all perform experiments based on their respective network models. First, they make 10 gestures, and each action lasts for 2 seconds. During this period, every 5 recognition results are obtained to make a judgment. The gesture with the most number of times for every 5 gesture results is regarded as a prosthetic hand control instruction. Every 10 gesture is a round, repeat the above experiment 15 times, rest for 5 minutes between each round, and do not move the position of the Myo armband during the whole experiment.

In the process of online gesture recognition, the 10 gestures correspond to codes 0~9, for example, “no. 1” corresponds to the code “0” and “first” corresponds to the code “6.” Then, the program will send the code of the experiment result to the intelligent prosthetic hand system. After receiving the instruction signal, the system will convert the signal into the rotation angle of the corresponding steering gear and finally realize the control of the intelligent prosthetic hand.

Figure 15 shows the status of gesture recognition and intelligent prosthetic hand control.

A total of 300 controls of the intelligent dummy hand were completed in this experiment.  Figure 16 records the number of experiments in which each of the 10 gestures was correctly recognized versus incorrectly recognized. The best recognition was achieved for the “first” and “good,” both of which were correctly recognized up to 29 times, which shows that the distinguishability of the “first” and “good” is higher compared to other gestures. However, no. 4 and no. 6 gestures have a lower recognizability. The reason may be that there are differences in the signal intensities acquired during the sEMG acquisition process, which affects the recognition effect of the system. Therefore, it is very necessary to conduct a unified muscle force training for the subjects before the experiment. Secondly, it may be due to the low degree of distinction between the various hand movements, which can easily be mistaken for other gestures similar to it.

To clearly see the effectiveness of the proposed MSFS-TCND method applied to real-time gesture recognition, in Table 7, we calculate the accuracy, recall, precision, and *F*1 score for online recognition of 10 gestures. The average online recognition accuracy of 10 gestures reaches 90.0%.

## 4. Conclusion

Due to the complex and ever-changing environment, the traditional way of controlling robots is gradually revealing its drawbacks. In order to improve the accuracy and efficiency of the control of the robot, this paper proposes a system based on sEMG to control the intelligent prosthetic hand. It can be applied in the field of rehabilitation robot and remote control robot.

The article proposes that the MSFS method can improve the richness of the acquired sEMG by adding virtual sEMG channels. In addition, the deep learning TCN is improved and combined with the MSFS method to improve the accuracy of gesture recognition. The test data demonstrates that the accuracy of real-time gesture recognition is substantially improved by combining MSFS with the improved TCN. Finally, in order to verify the validity of the proposed network, an intelligent robotic system based on 3D printing technology is designed. The intelligent prosthetic hand can accurately respond to the subject's movement intention.

In future research, try to include the feedback information of the intelligent prosthetic hand, so as to continuously improve the intelligent prosthetic hand system.

## Figures and Tables

**Figure 1:** The scheme of the entire process.

**Figure 2:** Data acquisition status of the gestures.

**Figure 3:** The operation of the MSFS method.

**Figure 4:** Comparison of sEMG signals before and after denoising.

**Figure 5:** The operation of sliding window.

**Figure 6:** Visual structure diagram of the expanded convolutional layer.

**Figure 7:** The TCNS architecture.

**Figure 8:** The TCND architecture.

**Figure 9:** Cumulative variance contribution rate of PCA dimension reduction.

**Figure 10:** Accuracy curves of the network training set for the proposed two TCN models.

**Figure 11:** Loss curves of the network training set for the proposed two TCN models.

**Figure 12:** Accuracy curve of network training set.

**Figure 13:** The hardware structure of prosthetic hand.

**Figure 14:** The implementation process of the system.

**Figure 15:** The status of intelligent prosthetic hand control.

**Figure 16:** Number of successes and failures in online gesture recognition.

**Table 1:** Subject information in the Myo_data dataset.

Number of subjects	Male to female ratio	Average height (cm)	Average weight (kg)	Average body mass index (kg/m^2^)
10	1 : 1	170.6 ± 9.49	62.19 ± 3.12	21.37 ± 3.28

**Table 2:** Specific information for 4 subjects.

Subject	Gender	Age	Height (cm)	Weight (kg)	Average body mass index (kg/m^2^)
A	Male	24	175	74	24.16
B	Female	23	165	55	20.20
C	Male	26	180	81	25.00
D	Female	24	155	50	20.81

**Table 3:** Pearson correlation coefficient.

Pearson correlation coefficient (average value)	Adjacent rows	Adjacent columns
*r*_NoMSFS_	0.47	0.42
*r*_MSFS_	0.29	0.39

**Table 4:** Dimensionality reduction results.

Database	Input dimension	The number of principal components
Myo_data	80	10
Myo_data+MSFS	160	20
DB5	160	20
DB5+MSFS	320	40

**Table 5:** The accuracy, recall, and precision of 10-gesture recognition (%).

Algorithm	MSFS (Y/N)	Dimension	Accuracy	Recall	Precision	*F*1 score
KNN	N	10	87.59	87.60	87.70	87.65
KNN	Y	20	88.63	88.64	88.70	88.67
LDA	N	10	87.67	87.68	87.85	87.76
LDA	Y	20	88.15	88.19	88.32	88.25
SVM	N	10	84.74	84.70	84.89	84.79
SVM	Y	20	85.27	85.24	85.42	85.33

**Table 6:** The average accuracy of 10-gesture recognition (%).

Algorithm	MSFS (Y/N)	Accuracy	Recall	Precision	*F*1 score
TCNS	N	91.52	91.54	91.60	91.57
TCNS	Y	92.34	92.36	92.42	92.39
TCND	N	92.41	92.44	92.61	92.52
TCND	Y	93.69	93.71	93.80	93.75

**Table 7:** Average accuracy (%) of 10-gesture recognition by applying MSFS-TCND algorithm.

Algorithm	Accuracy	Recall	Precision	*F*1 score
MSFS-TCND	90.03	90.25	90.11	89.97

## Data Availability

The program data used to support the findings of this study are available from the corresponding author upon request.
